# A Review on the Rule-Based Filtering Structure with Applications on Computational Biomedical Images

**DOI:** 10.1155/2022/2599256

**Published:** 2022-03-08

**Authors:** Xiao-Xia Yin, Sillas Hadjiloucas, Le Sun, John W. Bowen, Yanchun Zhang

**Affiliations:** ^1^Cyberspace Institute of Advanced Technology, Guangzhou University, Guangzhou 510006, China; ^2^Biomedical Engineering, School of Biological Sciences, University of Reading, Reading RG6 6AY, UK; ^3^Engineering Research Center of Digital Forensics, Ministry of Education, Nanjing University of Information Science and Technology, Nanjing, China

## Abstract

In this paper, we present rule-based fuzzy inference systems that consist of a series of mathematical representations based on fuzzy concepts in the filtering structure. It is crucial for understanding and discussing different principles associated with fuzzy filter design procedures. A number of typical fuzzy multichannel filtering approaches are provided in order to clarify the different fuzzy filter designs and compare different algorithms. In particular, in most practical applications (i.e., biomedical image analysis), the emphasis is placed primarily on fuzzy filtering algorithms, with the main advantages of restoration of corrupted medical images and the interpretation capability, along with the capability of edge preservation and relevant image information for accurate diagnosis of diseases.

## 1. Introduction

From a biomedical image reconstruction perspective, fuzzy filtering is particularly useful because it enables the denoising of extremely corrupted color images [1]. As a result, future knowledge-based systems for biomedical imaging are likely to incorporate fuzzy operators in their software [2]. Various noise forms impair color pictures in various approaches, and this poses a major challenge to the design of multichannel filters [3–6].

In order to successfully address the problem of color image denoising, the challenge is to (a) trace the origins and account for the diversity of the noise characteristics and (b) take into consideration the nonstationary statistics of the underlying image structures [7]. The above considerations have fueled current academic exertions aimed at merging structure or noise estimation approaches alongside filtering techniques regarding color image restoration. There are three main objectives that need to be fulfilled when designing filters for color image restoration: noise attenuation, chromaticity retention, and edge detail preservation [8].

Numerous signal processing issues, particularly those involving the nonlinearities of the picture creation process, cannot be successfully treated using linear approaches. Additionally, one must consider the human visual system's nonlinear nature [9]. Fuzzy modelling provides a bridge between linear and nonlinear techniques by integrating conventional linear and nonlinear filters with fuzzy logic. Since information extracted from data may also be corrupted by noise, a precise mathematic model of a nonlinear system is more difficult to establish because it requires a deterministic component in the model and a separate stochastic one, increasing the number of parameters that need to be evaluated. Fuzzy reasoning is particularly well suited from this perspective as it enables the choice of soft thresholds that can adapt better to the nonlinearities in the model inputs [9, 10].

The method of applying fuzzy logic to formulate a mapping to an output from a given input is fuzzy inference. This mapping then serves as a foundation for decision-making and pattern recognition [11]. In modelling, the fuzzy rule-based method considers orally defined rules that overlap in the parameter space [12, 13]. In the fuzzy modelling process, the aim is to derive a fuzzy rule base that is appropriate for the task at hand. As a fuzzy filter takes into account selected patterns in the neighbourhood of the element to be processed, the filtered output is capable of adapting to information present in the vicinity of the pixels being processed. To restore and correct a corrupted pixel locally, a window-based fuzzy filter is normally used, where the fuzzy rule acts directly on the signal elements within the operational window.

However, a significant number of rules is often needed, and the designer must strike a balance between rule count and performance because even a modest processing window frequently requires a huge number of rules [14]. To address these issues, data-dependent filters based on fuzzy reasoning have been developed. To derive fuzzy rules automatically, two fundamental problems concerning fuzzy system modelling should be addressed: one is fuzzy rule parameter optimization and the other is the identification of an appropriate system structure in relation to the number of membership functions and fuzzy rules [15]. A three-step approach is applied to achieve the fuzzy inference process; this involves the right choice of membership functions, fuzzy logic operators, and if-then rules [11].

Concluding, the basic motivation behind this work is not to elaborate into new ideas in fuzzy logic theory but to use effectively fuzzy logic techniques into the filtering of multidimensional data and color images with biomedical applications. The presented method can be generalized to any dimension and can be used effectively to other types of correlated multidimensional/multichannel data as well.

This paper is organized as follows.  Section 2 addresses the generation of suitable membership functions for fuzzy variables. Identification of optimized equation parameters through fuzzy rule modelling is also reviewed in this section.  Section 3 discusses the use of a membership function to restore the corrupted pixels in a color image.  Section 4 contains various fuzzy filter construction through fuzzy inferences.  Section 5 discusses how the fuzzy reduction approach may be used to analyze, restore, and repair biomedical imaging. Finally, Section 6 provides a concise summary of the most important aspects in each section.

## 2. Fuzzy Variables and Fuzzy Rules for a Color Image

It is widely accepted that color conveys additional information beyond that conveyed in greyscale imaging. As a result, color and multispectral imaging systems are used in most scientific applications. The origins of such advantage may be traced to Fellgett's multiplex advantage in astronomy, which states that a multispectral system has an advantage over its monochromatic counterpart because of higher throughput per unit time associated with the different separate channels conveying the acquired information. Within the context of acquiring information from different channels, noise filtering is one of the most common image processing tasks and forms an essential part of any image processing system [16, 17].

Instead of adopting traditional vector filters for a fixed amount of smoothing or noise removal [3], it is possible to adapt the smoothing criterion to local image statistics. Two basic assumptions play an important role in filtering techniques development [18]. One is that a noise-free image should be locally and smoothly varying while at the same time also separated by edges [19]. The other is that, normally, a noise pixel possesses a gray value that is much more or lesser than that of its neighbors [20]. Any fuzzy rule is associated with a local representation over a region defined in the input space [21]. A particular window, as illustrated in Figure 1, can thus be designed to define a region with pixels corrupted by impulse noise.

To design a fuzzy filter, it is important to clarify where and how a particular membership function arises, how it is used and its effect is quantified, and how it can be tailored according to the imaging problem at hand in order to provide meaningful results. Different interpretations of fuzziness result in a multiplicity of solutions to graded membership and membership definition problems [22]. The following sections review some basic concepts and defines fuzzy (logic) variables concerning color images. The adopted approaches to calculating specific fuzzy variables are represented as special cases tailored to specific problems. They lead to relevant membership functions suitable for achieving the outputs of the ruled fuzzy filters.

### 2.1. Adaptive Fuzzy Hybrid Approaches

The adaptive fuzzy hybrid multichannel (AFHM) filter [23] provides the generic framework that incorporates the ideas from the following three filters: the vector median (VM) filter, the vector directional (VD) filter, and the identity filter [23].

Let *d*_*VM*_ and *d*_*ξ*,*VM*_ denote the aggregated Euclidean distances corresponding to **y**_*VM*_ and **y**_*ξ*_ (the central vector-valued pixel), respectively. In addition, let *d*_*BV*  *D*_ and *d*_*ξ*,*BV*  *D*_ denote the aggregated angular distances corresponding to **y**_*BV*  *D*_ and **y**_*ξ*_, respectively. It is obvious that *d*_*VM*_ < *d*_*ξ*,*VM*_ and *d*_*BV*  *D*_ < *d*_*ξ*,*BV*  *D*_.

Let *μ* and *ν* denote two measures as fuzzy varieties for detecting the possibility whether the central vector-valued pixel is contaminated or not. A big *μ*-value suggests the substantial probability of contamination of the center vector-valued pixel. A big *ν*-value indicates the center vector-valued pixel's direction to be more possibly a directional outlier [24]. We define *μ* and *ν* as fuzzy varieties, which satisfy the following equations, respectively.

(1) $$\begin{array}{c} \mu =\left|d_{VM}-d_{\xi ,VM}\right|,\\ \nu =\left|d_{BV\;D}-d_{\xi ,BV\;D}\right|. \end{array}$$

When both *μ* and *ν* are large, this indicates that the chance of corrupting the center vector-valued pixel **y**_*ξ*_ is significantly high. The aggregated distance between a corrupted vector-valued pixel and the median vector should be large [23]. When only *μ* is small, this indicates that **y**_*ξ*_ is regarded as an uncorrupted vector by the VM filter but a corrupted vector by the BVD filter. When only *ν* is small, the situation is opposite. When both *μ* and *ν* are small, there is high possibility that the center pixel is not corrupted by noise.

### 2.2. Applications of the Fuzzy Derivative

It has been shown that fuzzy derivatives are useful for fuzzy filtering. A simple derivative at the central pixel position (*k*_1_, *k*_2_) in the direction **D**(**D***ɛ ***DIR**={**NW**, **W**, **SW**, **S**, **SE**, **E**, **NE**, **N**}) is defined as the difference between the pixel at (*k*_1_, *k*_2_) and its neighbor in the direction **D**. This derivative value is denoted by ∇_**D**_(*k*_1_, *k*_2_). This can be expressed as follows:

(2) $$\begin{array}{c} \nabla_{D}\left(k_{1},k_{2}\right)=x\left(k_{1}-1,k_{2}-1\right)-x\left(k_{1},k_{2}\right). \end{array}$$

The fuzzy derivative's principal idea considers this observation. Assume an edge that runs in the **SW** − **NE** direction across the neighborhood of a pixel (*k*_1_, *k*_2_). The derivative gains a big value. Additionally, the derivative values of nearby pixels perpendicular to the direction of the edge might be rather considerable. To carry out the edge detection procedure, one basic gradient value and two associated gradient values (specified in the same direction) are generated for each direction. These correspond to the two parameters ∇_**D**_(*k*_1_, *k*_2_), ∇_**D**_(*k*_1_+1, *k*_2_ − 1), ∇_**D**_(*k*_1_ − 1, *k*_2_+1), respectively; see Figure 1(b). The objective is to cancel out the influence of a single high derivative value caused by noise. Thus, if two of the three derivative values are small, it is generally reasonable to believe that the considered direction lacks an edge. The stated assumption is considered when the fuzzy rule for computing fuzzy derivative values is developed [25]. For an overview of how the pixels are used to calculate the fuzzy derivative for each direction, one can refer to [25].  Figure 1(a) illustrates the neighborhood of a central pixel (*k*_1_, *k*_2_). In Figure 1(b), pixel values indicated in gray are used to compute the “fuzzy derivative” of the central pixel (*k*_1_, *k*_2_) for the NW-direction [25].

In [26], the fuzzy gradient (derivative) value, associated with a noisy component of a center pixel (e.g., the red component), ∇_*D*_^*F*^*C*_*R*_(*k*_1_, *k*_2_) can be defined according to a fuzzy fusion function which has a span between the basic gradient value and the two related gradient values in the direction *D*.

(3) $$\begin{array}{c} \nabla_{D}^{F}C_{R}{\left(k_{1},k_{2}\right)}^{\text{noise}}\\ ={\left|\nabla_{D}C_{R}\left(k_{1},k_{2}\right)\right|}^{S}\cap {\left|{\dot{\nabla }}_{D}C_{R}\left(k_{1},k_{2}\right)\right|}^{L}\cap {\left|{\overset{..}{\nabla }}_{D}C_{R}\left(k_{1},k_{2}\right)\right|}^{L}\cup {\left|\nabla_{D}C_{R}\left(k_{1},k_{2}\right)\right|}^{L}\cap {\left|{\dot{\nabla }}_{D}C_{R}\left(k_{1},k_{2}\right)\right|}^{S}\cup {\left|{\overset{..}{\nabla }}_{D}C_{R}\left(k_{1},k_{2}\right)\right|}^{S}. \end{array}$$

This way, it is possible to obtain the fuzzy gradient (derivative) value regarding the free noisy (red) component of a center pixel in the direction *D*.

(4) $$\begin{array}{c} \nabla_{D}^{F}C_{R}{\left(k_{1},k_{2}\right)}^{\text{noisefree}}\\ ={\left|\nabla_{D}C_{R}\left(k_{1},k_{2}\right)\right|}^{L}\cap {\left|{\dot{\nabla }}_{D}C_{R}\left(k_{1},k_{2}\right)\right|}^{L}\cap {\left|{\overset{..}{\nabla }}_{D}C_{R}\left(k_{1},k_{2}\right)\right|}^{L}\cup {\left|\nabla_{D}C_{R}\left(k_{1},k_{2}\right)\right|}^{S}\cap {\left|{\dot{\nabla }}_{D}C_{R}\left(k_{1},k_{2}\right)\right|}^{S}\cap {\left|{\overset{..}{\nabla }}_{D}C_{R}\left(k_{1},k_{2}\right)\right|}^{S}. \end{array}$$

The sign ∇_*D*_*C*_*R*_(*k*_1_, *k*_2_) is the basic gradient value (for the red component); ${\dot{\nabla }}_{D}C_{R}\left(k_{1},k_{2}\right)$ and ${\overset{..}{\nabla }}_{D}C_{R}\left(k_{1},k_{2}\right)$ are the two related gradient values in the direction *D*. The fuzzy sets *large* and *small* are denoted as |*·*|^*L*^ and |*·*|^*S*^, respectively.

The fuzzy gradient (derivative) value regarding the noisy red component of a center pixel, ∇_*D*_^*F*^*C*_*R*_(*k*_1_, *k*_2_) can also be defined using a fuzzy set *large*, *small*, *big positive* and *big negative*, denoted as |.|^*L*^ and |·|^*S*^, respectively.

(5) $$\begin{array}{c} \nabla_{D}^{F}C_{R}{\left(k_{1},k_{2}\right)}^{L}\\ ={\left|\nabla_{D}C_{R}\left(k_{1},k_{2}\right)\right|}^{L}\cap {\left|{\dot{\nabla }}_{D}C_{R}\left(k_{1},k_{2}\right)\right|}^{S}\cup {\left|\nabla_{D}C_{R}\left(k_{1},k_{2}\right)\right|}^{L}\\ \cap {\left|{\overset{..}{\nabla }}_{D}C_{R}\left(k_{1},k_{2}\right)\right|}^{S}\cup {\left|\nabla_{D}C_{R}\left(k_{1},k_{2}\right)\right|}^{BP}\cap {\left({\dot{\nabla }}_{D}C_{R}C_{R}\left(k_{1},k_{2}\right)\cap {\overset{..}{\nabla }}_{D}C_{R}\left(k_{1},k_{2}\right)\right)}^{BN}\\ \cup \nabla_{D}C_{R}C_{R}{\left(k_{1},k_{2}\right)}^{BN}\cap {\left({\dot{\nabla }}_{D}C_{R}C_{R}\left(k_{1},k_{2}\right)\cap {\overset{..}{\nabla }}_{D}C_{R}\left(k_{1},k_{2}\right)\right)}^{BP}. \end{array}$$

Further details on the formulation of these fuzzy sets can be found in [27].

Using fuzzy rules, the red component of a central pixel *C*_*R*_(*k*_1_, *k*_2_) can therefore be identified as being corrupted with impulse noise, if more than half of the fuzzy gradient values (more than four for a nonborder placed pixel) are part of a *α* ∈ (0,1] (weak) level of the fuzzy set *large* [28]. The application of local directional gradients using fuzzy logic to detect an outlier pixel and calculate the outputs of such a fuzzy filter is also discussed by [9].

The fuzzy derivative method mentioned above can be used to achieve perform uniformly distributed (random valued) impulse noise detection [26, 27]. Another approach for identifying random valued impulse noise pixels is to investigate the state of the neighborhood around a pixel. The detection process requires the construction of suitable fuzzy sets' *noise* for each color component at each position of an image [26, 27]. This method achieves random valued impulse noise detection.

In the current method, the mean difference in a *H* × *S* window denoted as *g*(*k*_1_, *k*_2_) is calculated:

(6) $$\begin{array}{c} g\left(k_{1},k_{2}\right)=\frac{\sum_{h=-H}^{H}\sum_{s=-S}^{S}\left|x\left(k_{1}+h,k_{2}+s\right)-x\left(k_{1},k_{2}\right)\right|}{\left(2H+1\right)\left(2S+1\right)-1}. \end{array}$$

Corrupted impulse noise pixels generally cause large *g*(*k*_1_, *k*_2_) values because impulse noise pixels normally occur as outliers in a small neighborhood around the pixel. On the other hand, the *g*(*k*_1_, *k*_2_) value could be relatively large in the case of an edge pixel. Therefore, the following two values denoted as obs_1_(*k*_1_, *k*_2_) and obs_2_(*k*_1_, *k*_2_) are considered:

(7) $$\begin{array}{c} {\text{obs}}_{1}\left(k_{1},k_{2}\right)=\frac{\sum_{h=-H}^{H}\sum_{s=-S}^{S}g\left(k_{1}+h,k_{2}+s\right)}{\left(2H+1\right)\left(2S+1\right)}, \end{array}$$

(8) $$\begin{array}{c} {\text{obs}}_{2}\left(k_{1},k_{2}\right)=g\left(k_{1}+h,k_{2}+s\right). \end{array}$$

If both values obs_1_(*k*_1_, *k*_2_) and obs_2_(*k*_1_, *k*_2_) are large, then the pixel can be considered as an edge pixel instead of a noisy one. So, when the two values obs_1_(*k*_1_, *k*_2_) and obs_2_(*k*_1_, *k*_2_) are very similar, it is concluded that the pixel is noise free. Otherwise, if the difference between obs_1_(*k*_1_, *k*_2_) and obs_1_(*k*_1_, *k*_2_) is large, then the pixel is considered as noisy.

Agrawal et al. [29] conducted fuzzy derivative and fuzzy smoothing based on fuzzy rules, which make use of membership functions for removal of narrow-tailed and medium narrow-tailed noise in medical images. Iteratively applying the filter significantly reduces background noise. The form of the membership functions is modified depending on the residual level of noise following every iteration, taking use of the image's homogeneity distribution. A statistical model for noise distribution may be used to connect the homogeneity of the membership functions to their adaptation method. Experiments are conducted to demonstrate the practicality of the suggested technique. Additionally, these findings are compared to those obtained from other filters using numerical metrics and ocular examination.

In addition, Ma et al. [4] proposed an improved version of the partition filter that takes advantage of partition-based trimmed vector median, instead of center-weighted vector median as a fuzzy reference estimate can be considered. Partition-based trimmed vector median is different from center-weighted trimmed vector median in that the latter replaces the threshold value of center-weighted trimmed vector median with (*N* − 1)/2. The resultant algorithm of this improved version of the fuzzy partition filter simplifies computation and adapts well to the local properties of image structures.

As an important extension of fuzzy derivative, the fuzzy *n*th-order derivative and fuzzy differential equations of fractional order using Laplace and integral transforms are investigated by Ahmadi et al. [30] and Salahshour et al. [31], respectively. The most important advantage of this fuzzy differential procedure is the significantly reduced computational complexity in dealing with the fractional/*n*th-order derivative.

## 3. Membership Function

One of the most difficult aspects of designing fuzzy systems is generating appropriate fuzzy variables' membership functions [32]. A fuzzy constraint to single parameter is normally defined by a fuzzy membership function with values within [0,1] [33]. Each response input and output has a unique membership function.

Generally, the membership function *μ*_*𝒜*_(*x*) describes the membership of the elements *x* of the base set *𝒳* in the fuzzy set *𝒜*, whereby for *μ*_*𝒜*_(*x*) a large class of functions can be taken assumed. In other words, a fuzzy set is formed on the basis of a membership function that generates the membership degree [34]; this enables the progressive evaluation of the membership of set components [35].

Membership functions with reasonable membership are typically piecewise linear functions, including trapezoidal or triangular functions. Certain applications require continuously differentiable curves and, consequently, smooth transitions. Smoothness is often achieved using Gaussian and other bell-shaped membership functions. In addition, for certain applications, it is also important to define asymmetric membership functions. Asymmetric and closed sigmoidal membership functions can be generally synthesized using two sigmoidal functions.

For many other applications, these membership functions mentioned above are insufficient because they are not accurately representative of the linguistic terms being modelled; thus, they must be elicited directly from experts, either through a “statistical” way or through an automatic generation of specific pass- and reject-band filter shapes. This is an emergent topic in the current artificial intelligence literature, as the aim is to develop automated fuzzy inference engines. Before discussing such approaches, however, it is worthwhile to consider traditional (manual) approaches.

### 3.1. Similarity Measurements

Consideration of membership values as similarity indicators is typically utilized in prototype theory, where membership is defined as the state of being similar to a category's representative [36]. Therefore, a membership function value may be utilized to measure an element's degree of resemblance to a given set [22].

#### 3.1.1. Adaptive Color Pixel Similarity Function

Based on [7], in robust signal processing, sample rank ordering is often utilized. Recent breakthroughs in fuzzy set theory have integrated sample rank ordering in the temporal domain or the spatial ordering of observations [37–41]. Given two color pixels, *x* and *y*, there exists a wide range of functions [5, 17, 38, 42, 43], *μ*(*x*, *y*), which can be used to assess their physical similarity and meet the constraints of a fuzzy membership function; that is,

- *μ*(**x**, **y**)⟶1 if ‖**x** − **y**‖⟶0
- *μ*(**x**, **y**)⟶0 if ‖**x** − **y**‖⟶*∞*
- *μ*(**x**_1_, **y**_1_) ≥ *μ*(**x**_2_, **y**_2_), ∀‖(**x**_1_ − **y**_1_) ≥ ‖**x**_2_ − **y**_2_‖

The objective is to choose an acceptable Gaussian function to express similarities between two color pixels, which is facilitated by the exponential nature of perceptual distance measurements [5, 44]. The ideal sample spread associated with each kind of Gaussian function may be determined using the mean absolute error (MAE) criteria as described in [45]. Additionally, in [7, 46], a resolution to noise deviation estimates is proposed. This strategy is used in [7], which compares two different forms of Gaussian functions. The first is a scalar Gaussian function *μ*_1_ based on the vectors' Euclidean distance, and the second is a vector of component-wise Gaussian functions *μ*_2_ in the YCbCr or RGB color space. Compared to the simpler *μ*_1_ scalar function, the *μ*_2_ function provides additional flexibility in modelling the similarity membership, but its performance in various color spaces is weak in the RGB space, running a risk of an expensive computation cost due to its component-wise sample spread. As new expanded color spaces are introduced by industry, this can be an interesting approach.

#### 3.1.2. A Self-Adaptive Algorithm

A new way of defining the similarity function is introduced in [17]. There is an attempt to achieve nonascending, *convex* similarity measures, with the use of a natural normalization of the similarity function, satisfying *μ*(0)=1, *μ*(*∞*)=0.

The *convex* membership functions for the similarity measures can be treated as kernels of nonparametric density estimation, as illustrated in [17, 47, 48]. The expression in (10) is shown to be particularly effective as discussed in [17, 49, 50].

(9) $$\begin{array}{c} \mu \left(x_{i},x_{j}\right)=\left\{\begin{array}{cc} 1, & -\frac{\rho \left(x_{i},x_{j}\right)}{h}\text{ for }\rho \left(x_{i},x_{j}\right)<h,\\ 0, & \text{otherwise}, \end{array}\right. \end{array}$$

where *ρ*{**x**_*i*_, **x**_*j*_}=‖**x**_**i**_ − **x**_**j**_‖.

The parameter *h* is determined on the basis of the image structure and noise statistics. It influences the severity of the filtering process so that a decreasing function of *h* related to the fraction of pixels is replaced. Compared with the vector median filter (VMF), corresponding to *h*=0, the resultant filter shows enhanced performance. Performance can be tuned by specifying positive values of *h*, compelling the filter to maintain uncorrupted original pixels to a greater or lesser extent, while still enabling the removal of corrupted ones.

Using the **L**_2_ norm of the Euclidean distance between two pixels in the RGB color space, it is possible to estimate the fraction of corrupted pixels. Thus, among eight neighboring pixels around a center pixel, there exists at least *m* pixels that have a **L**_2_ norm less than a predefined constant *d*.

#### 3.1.3. Fuzzy Color Correlation

An alternative approach to traditional vector-based approaches is the idea by [51], which achieves similarity measurements in each color component between the central pixel **x**_0_ and each color neighbour **x**_*k*_, separately, the approach also assesses whether the local differences in one, for example, the *R* component, neighborhood corresponds to the differences found in the *G* and *B* components. We denote these two memberships with *S*_1_ and *S*_2_.

The aim is to first to develop membership function that may be used to check these differences of neighbor component, which can be represented through a fuzzy set *small*.

(10) $$\begin{array}{c} 1-S\left(x\right)=S_{1}=\left\{\begin{array}{cc} 1, & x\leq \alpha_{1},\\ 1-2{\left(\frac{x-\gamma_{1}}{\gamma_{1}-\alpha_{1}}\right)}^{2}, & \alpha_{1}<x<\frac{\alpha_{1}+\gamma_{1}}{2},\\ 2{\left(\frac{x-\gamma_{1}}{\gamma_{1}-\alpha_{1}}\right)}^{2}, & \frac{\alpha_{1}+\gamma_{1}}{2}<x<\gamma_{1},\\ 0, & x>\gamma_{1}, \end{array}\right. \end{array}$$

where *α*_1_=10 and *γ*_1_=70 can achieve experimentally satisfying results of noise filtering. The second item element of equation (10) shows a large membership degree with a relatively small difference and a slow decrease in the membership degree. The third item element is a parameter used to decrease the membership degree faster for each larger difference after a certain point. As a result, the membership function defined in equation (10) is also utilized to calculate the absolute value of the membership degree differences in the fuzzy set *S*_1_ for the green and red components, as well as the blue and red components. If one denotes the relevant membership function as *S*_2_, the membership function equation (10) is calculated, with *α*_1_=0.01 and *γ*_1_=0.15.

A further interest in this work is that it enables the identification of noise-free center pixels in a different color channel. The noise-free degree of *x*_0_^*R*^, denoted as *NF*_*x*_0_^*R*^_, is calculated as follows by utilizing the product triangular norm representing both the fuzzy OR (disjunction) operator and the fuzzy AND (conjunction) operator.

(11) $$\begin{array}{c} NF_{x_{0}^{R}}=\mu^{R}\mu^{RG}\mu^{G}+\mu^{R}\mu^{RB}\mu^{B}-\mu^{R}\mu^{RG}\mu^{G}\mu^{R}\mu^{RB}\mu^{B}, \end{array}$$

where the standard negation operation is used to derive the membership degree in the fuzzy set *noise free* for each color component. Here, *μ*^*R*^ and *μ*^*RG*^ are the conjunction of *S*_1_(Δ*F*_*k*_^*R*^) and *μ*_*k*_^*RG*^ in the distance measurement of a red component and the difference between the membership degrees in the fuzzy set *S*_1_ for the red and the blue components. A similar computation can be performed for the other color components. The noise-free degrees of blue *NF*_*x*_0_^*B*^_ and green *NF*_*x*_0_^*G*^_ components of the center pixel can thus be achieved.

### 3.2. Histogram-Based Approaches

In order to establish connections among different smaller membership functions, in [52], it is proposed to calculate the slope difference of each selected intensity value from a color image. This approach uses the histogram approach described earlier to establish a separate membership function (denoted as *μ*_noise_*p*^*k*^__). Given each selected integer value *p*^*k*^, the membership function can be expressed as follows:

(12) $$\begin{array}{c} \mu_{{\text{noise}}_{p_{k}}}\left\{\begin{array}{cc} 0, & \left(\forall x\leq a_{k}\right)\text{ or }\left(\forall x\geq d_{k}\right),\\ 2{\left(\frac{x-a_{k}}{b_{k}-a_{k}}\right)}^{2}, & \forall x\in \left(a_{k},\frac{a_{k}-b_{k}}{2}\right],\\ 1-2{\left(\frac{x-b_{k}}{b_{k}-a_{k}}\right)}^{2}, & \forall x\in \left(\frac{a_{k}+b_{k}}{2},b_{k}\right),\\ 1, & \forall x\geq \left[b_{k},c_{k}\right],\\ 1-2{\left(\frac{x-c_{k}}{d_{k}-c_{k}}\right)}^{2}, & \forall x\in \left(c_{k},\frac{c_{k}+d_{k}}{2}\right],\\ 2{\left(\frac{x-d_{k}}{d_{k}-c_{k}}\right)}^{2}, & \forall x\in \left(\frac{c_{k}+d_{k}}{2},d_{k}\right). \end{array}\right. \end{array}$$

The membership function *impulse noise* (for the red component) *μ*_impulse_^*R*^ then becomes

(13) $$\begin{array}{c} \mu_{\text{impulse}}\left(C_{R}\left(k_{1},k_{2}\right)\right)=\underset{k\in \left\{1,\ldots ,n\right\}}{\max}\mu_{\mathrm{noise}/p_{k}}\left(C_{R}\left(k_{1},k_{2}\right)\right). \end{array}$$

The parameters used in expression (13) are related to the slope of each the selected intensity value. There exist two different types of noise histograms. The histograms containing only peaks normally have a very small slope and the histograms containing peaks with some other features normally have a larger slope. These are treated as a relation with the low estimated standard deviation and large estimated standard deviation, respectively. Based on the edge image produced by the Sobel operator [53], the following expressions are proposed to calculate these parameters:

(14) $$\begin{array}{c} a_{k}=p^{k}-\vartheta_{a},\\ b_{k}=p^{k}-\vartheta_{b},\\ c_{k}=p^{k}+\vartheta_{c},\\ d_{k}=p^{k}+\vartheta_{d},\\ \vartheta_{b}=\frac{2}{3\vartheta_{a},},\\ \vartheta_{c}=\frac{2}{3\vartheta_{d}}\\ \vartheta_{a}=\vartheta_{d}=\min\left(25,\left\lfloor \sigma \right\rfloor \right), \end{array}$$

where ⌊*σ*⌋ is the largest integer value that is smaller than the standard deviation (variance) *σ*. This method of parameter selection is especially well suited for denoising pictures that have been damaged by a combination of impulse and Gaussian noise. When ⌊*σ*⌋>20, to prevent overfiltering, *ϑ*_*a*_ and *ϑ*_*d*_ are then restricted to be a value of 20. Further discussion regarding the histogram based methods can be found in [26].

Based on [26], with existing fixed-value impulse noise, histograms are initially created from most likely corrupted impulse noise color components. Since pixels that have been damaged by fixed-value impulse noise are often very dissimilar to their neighbors, they are usually identified in a local window by their minimum and maximum intensity values, denoted as *p*_max_ or *p*_min_. In order to calculate histograms for each image component, a two-step process is involved: (a) the corrupted greyscale images are divided into small blocks from each color channel, with a suggested block size of 5 × 5; and (b) the determination of the values of the two intensity levels *p*_max_ or *p*_min_ to be adopted for the calculation of the histogram depends on the following conditions being simultaneously satisfied:

- If *p*_max_ is involved, then |*m*_1_ − *p*_max_| > |*m*_1_ − *m*_2_| or |*m*_2_ − *p*_max_| > |*m*_1_ − *m*_2_|
- If *p*_min_ is involved, then |*m*_1_ − *p*_min_| > |*m*_1_ − *m*_2_| or |*m*_2_ − *p*_min_| > |*m*_1_ − *m*_2_|
- Defining the membership degrees *μ*^noise^(*p*_*R*_) for the intensity value *p*_*R*_^*k*^ of a red component in the fuzzy set *noise*, if (*h*_*R*_^noise^(*k*)/∑_*l*=0_^255^*h*_*R*_^noise^(*l*)), then *k* is a noise red intensity

In the case of fixed-value impulse noise, at least a single intensity value with a membership degree of one in the fuzzy set *noise* is anticipated; or else, the picture is not damaged by fixed-value impulse noise. The random valued impulse noise detection technique does not need to be used in this circumstance.

In the case of a random valued impulse noise, the color difference, between, for example, the red and green components, in each direction *D* of this window around the center position is calculated and denoted as ϱ_RG_^*D*^. For each color difference ϱ_RG_^*D*^, *D* ∈ [1,8], bell-shaped membership functions are defined as *η*_small_, *η*_medium_, and *η*_large_ that represent the degree of membership in the corresponding fuzzy sets *small*, *medium*, and *large*:

(15) $$\begin{array}{c} \eta_{\mathrm{small}}\left(\varrho_{\text{RG}}^{D}\right)=\left\{\begin{array}{cc} 1, & \text{if }\varrho_{\text{RG}}^{D}\leq c_{1},\\ \frac{1}{1+{\left(\varrho_{\text{RG}}^{D}-c_{1}/a_{1}\right)}^{2}b_{1}}, & \text{if }\varrho_{\text{RG}}^{D}>c_{1}k=1,2,\ldots ,9. \end{array}\right.\\ \eta_{\text{medium}}\left(\varrho_{\text{RG}}^{D}\right)=\frac{1}{1+{\left(\varrho_{\text{RG}}^{D}-c_{2}/a_{2}\right)}^{2}b_{2}},\;k=1,2\text{,}\ldots ,9,\\ \eta_{\text{small}}\left(\varrho_{\text{RG}}^{D}\right)=\left\{\begin{array}{cc} \frac{1}{1+{\left(\varrho_{\text{RG}}^{D}-c_{3}/a_{3}\right)}^{2}b_{3}}, & \text{if }\varrho_{\text{RG}}^{D}\leq c_{3}k=1\text{,}2\text{,}\ldots ,9,\\ 1, & \text{if }\varrho_{\text{RG}}^{D}>c_{3}. \end{array}\right. \end{array}$$

Histogram adaptive filtering in [54, 55] is applied to achieve a solution to the parameter space. The parameters *b*1=*b*2=*b*3=17 are adopted and experimentally validated. They are set to be excessively larger than *c*_1_, *c*_2_, and *c*_3_, respectively, in order to adaptively filter out impulsive noise by the membership functions. The calculation of the parameters (*a*1, *c*1), (*a*2, *c*2), and (*a*3, *c*3) takes advantage of statistics of the estimated histograms, in relation to intensity differences between red and green values. The calculation of the parameters for the other color differences is very similar. The following calculations of fuzzy sets regarding centroids *small* (denoted as *CEN*_small_^RG^), *medium* (denoted as *CEN*_medium_^RG^), and *large* (denoted as *CEN*_large_^RG^) are the functions of the total histogram *h*_*RG*_, and two divided histograms *P*  *DF*_part_1__^*RG*^ and *P*  *DF*_part_2__^*RG*^ by the splitting point *M*=[2(2^*m*^ − 1)*·CEN*_medium_^RG^ − (2^*m*^ − 1)], where [*x*] is the largest integer value smaller than *x*.

(16) $$\begin{array}{c} {\text{PDF}}^{\text{RG}}\left(z\right)=\frac{h_{RG}\left(z\right)}{\sum_{k=-\left(2^{m}-1\right)}^{2^{m}-1}h_{\text{RG}}\left(k\right)},\\ CEN_{\text{medium}}^{RG}\left(z\right)=\sum_{k=-\left(2^{m}-1\right)}^{2^{m}-1}\frac{k}{2^{m+1}-1}P\;DF_{\text{RG}}\left(k\right),\\ CEN_{\text{small}}^{\text{RG}}\left(z\right)=\sum_{k=-\left(2^{m}-1\right)}^{M}\frac{k}{2^{m+1}-1}P\;DF_{\text{part}1}^{\text{RG}}\left(k\right),\\ CEN_{\text{large}}^{\text{RG}}\left(z\right)=\sum_{k=M+1}^{2^{m}-1}\frac{k}{2^{m+1}-1}P\;DF_{\text{part}2}^{\text{RG}}\left(k\right), \end{array}$$

where *P*  *DF*_RG_(*z*) is the potential density function of the histogram *h*_RG_ for index *z*(*z* ∈ [−(2*m* − 1), 2*m* − 1]) (with *m*being the amount of bits used to store a single intensity value (mostly *m*=8)). The index *k* varies from 1 to *H* × *S* in order to select one of the window values.

The calculation of the mass that corresponds to the support of a fuzzy set is a function of the subdivided histogram *h*_*RG*_ with three equal parts.

(17) $$\begin{array}{c} {\text{MASS}}_{\text{small}}^{\text{RG}}=\frac{\sum_{k=-\left(2^{m}-1\right)}^{M_{1}}h_{RG}\left(k\right)}{\sum_{k=-\left(2^{m}-1\right)}^{2^{m}-1}h_{RG}\left(k\right)},\\ {\text{MASS}}_{\text{medium}}^{\text{RG}}=\frac{\sum_{k=M_{1}+1}^{M_{2}}h_{RG}\left(k\right)}{\sum_{k=-\left(2^{m}-1\right)}^{2^{m}-1}h_{\text{RG}}\left(k\right)},\\ {\text{MASS}}_{\text{large}}^{RG}=\frac{\sum_{k=M_{2}+1}^{2^{m}-1}h_{\text{RG}}\left(k\right)}{\sum_{k=-\left(2^{m}-1\right)}^{2^{m}-1}h_{\text{RG}}\left(k\right)}, \end{array}$$

where *M*_1_=[2(2^*m*^ − 1)*·*CEN_medium_^RG^+CEN_small_^RG^/2 − (2^*m*^ − 1)] and *M*_2_=[2(2^*m*^ − 1) · (CEN_medium_^RG^+CEN_large_^RG^/2) − (2^*m*^ − 1)].

The values MASS and CEN obtained from the estimated histogram *h*_RG_ are, respectively, used for the parameters *a* and *c*, with *c*_1_=CEN_SMALL_^RG^, *c*_2_=CEN_MEDIUM_^RG^ , *c*_3_=CEN_LARGE_^RG^ and *a*_1_=MASS_SMALL_^RG^ , *a*_2_=MASS_MEDIUM_^RG^ , *a*_3_=MASS_LARGE_^RG^. Thus, the membership functions are completely specified.

The procedure of the histogram estimation *h*_*RG*_ can be used to estimate the histograms of all the other color differences (red-green, red-blue, and green-blue). The histogram estimation ranges between −255 and +255. Each red-green difference (i.e., *RG*(*i*, *j*)), for example, is included in the histogram *h*_RG_ if and only if the membership degree in the fuzzy set noise for both components is zero, in other words if *μ*_noise_(*C*_*R*_(*i*, *j*))=0 and *μ*_noise_(*C*_*G*_(*i*, *j*))=0.

The fuzzy set *noiseμ*_noise_ is represented by a membership degree as follows:

(18) $$\begin{array}{c} \mu_{\text{noise}}\left(C_{R}\left(i,j\right)\right)=\left\{\begin{array}{cc} \eta_{\text{noise}}\left(C_{R}\left(i,j\right)\right), & \text{if }{\text{cond}}_{1},\\ 0, & \text{otherwise,} \end{array}\right. \end{array}$$

with

(19) $$\begin{array}{c} {\text{cond}}_{1}=\sum_{D\in \left\{N,\ldots ,S\right\}}\tau_{\text{noise}}^{D}\geq \tau_{\text{free}}^{D}. \end{array}$$

The overall membership degrees to the fuzzy sets *τ*_noise_^*D*^(*C*_*R*_(*i*, *j*)) and *τ*_noise_^*D*^(*C*_*R*_(*i*, *j*)) are calculated on the basis of the eight membership degrees in the relevant fuzzy sets *impulse noise-free* for the eight directions around a certain central pixel position (*i*, *j*), respectively. The membership function of a fuzzy set *τ*_noise_(*C*_*R*_(*i*, *j*)) is illustrated in Figure 2. The parameters *a* and *b* are equal to

(20) $$\begin{array}{c} a=\frac{\left(\sum_{h=-H}^{H}\sum_{s=-S}^{S}g\left(k_{1}+h,k_{2}+s\right)\right)-g\left(k_{1},k_{2}\right)}{\left(2H+1\right)\left(2S+1\right)-1}, \end{array}$$

where *g* satisfies (6).

(21) $$\begin{array}{c} b=1.2a. \end{array}$$

The standard negator *N*_*s*_(*x*)=1 − *x* is used to calculate a fuzzy set *impulse noise-free*.

If cond_1_ is satisfied, the membership function *η*_noise_(*C*_*R*_(*i*, *j*)) has a similar shape to Figure 2, but with min_*h*∈{−*H*,…,*H*};*s*∈{−*S*,…,*S*}_*g*(*i*+*h*, *j*+*s*). This is used to define a central pixel *C*_*R*_(*i*, *j*) with fuzzy set *large*, and define *η*_noise_; that is, *η*_noise_(*C*_*R*_(*i*, *j*))=*μ*_large_(obs_1_ − obs_2_). In this figure, the horizontal axis corresponds to all possible differences between obs_1_ and obs_2_. Detailed explanation regarding (obs_1_ − obs_2_) can be found in equations (7) and (8).

The most homogeneous region around *C*_*R*_(*i*, *j*) results in the *g*(*i*+*k*, *j*+*l*) value, which corresponds to *a*. This region has the smallest amount of impulse-noise corrupted pixels. Experimental results have shown that the best choice for parameter *b* is *b*=1.2*a*, the larger the parameter *a*is, the larger the uncertainty interval (*a*, *b*) should be.

Several fuzzy rules are used in the aforementioned algorithm:

(i) Membership degrees for the elements ϱ_RG_^*D*^ in the fuzzy set *noise-free*:
    IF (*C*_R*D*_ is not noise) AND ((*C*_R*D*_ is not noise)
    THEN ϱ_RG_^*D*^ is noise-free
(i) A corrupted central pixel *C*_*R*_(*i*, *j*) with impulse noise:

  IF obs_1_ − obs_2_ is large
  THEN the central pixel *C*_*R*_(*i*, *j*) is an impulse noise pixel

Two additional fuzzy rules related to the central pixel *C*_*R*_(*i*, *j*) that is defined as an *impulse noise* and *impulse free* pixel in the direction *D* are represented in equations (3) and (4). The other two noise-corrupted color channels have analogous fuzzy rules. The second fuzzy rule can be transferred used to calculate the third via fuzzy rule from the evaluation of the relevant histograms.

Histogram-based fuzzy color filter is particularly effective for reducing high-impulse noise in digital images while preserving edge sharpness. Different from applying a greyscale algorithm on each color component separately, vector-based filtering methods can overcome artefacts introduced especially on edge or texture pixels when dealing with noisy color images [26]. The major improvement achieved by the histogram-based fuzzy color filter (HFC) is demonstrated in Figure 3. This figure illustrates the visual performance of a magnified part of the “Lena” image with 20% salt-and-pepper noise. It is clearly observed that HFC shows the best performance in the noise removal and detail preservation; meanwhile, it does not introduce new colors (especially in texture elements of an image) in contrast to many of the compared filters, including the fuzzy impulse noise detection and reducing method (FIDRM), the adaptive-weighted fuzzy mean filter (AWFM) from [56], the histogram adaptive fuzzy filter (HAF), dual-step fuzzy inference ruled by else-action filter (DSFIRE) [57], the tristate median filter (TSM) from [58], and vector mean filter (VMF). An objective evaluation is performed using the peak signal-to-noise ratio (PSNR) (Figure 4).

### 3.3. Fuzzy Peer Group-Based Algorithms

Following the traditional *peer group* filters, the authors in [59] claim that traditional methods adopt crisp ways to calculate distance threshold *d*; however, the similarity measurements are not that easy. Furthermore, the number of peer group members is determined using Fisher's linear discriminant (FLD), which often turns out not to be a desired peer group since more than the necessary number of clusters is always obtained.

To overcome this problem, a similarity membership function *μ* is introduced:

(22) $$\begin{array}{c} \mu_{1}\left(x_{i},x_{j}\right)=e^{-\left(\left\|x_{i}-x_{j}\right\|/\Psi \right)},\;\text{for }i,j=\left\{0,\ldots ,n^{2}-1\right\}, \end{array}$$

where Ψ > 0 is a fuzzy matrix [60, 61], and *μ*_1_=1 if **x**_0_=**x**_(*i*)_ so that

*μ*_1_(**x**_0_, **x**_(0)_) ≥ *μ*_1_(**x**_0_, **x**_(1)_) ≥ ⋯≥*μ*_1_(**x**_0_, **x**_(*n*^2^ − 1)_). And an accumulated similarity (fuzzy distance) metric *d*_PG_(**x**_0_, **x**_(*i*)_) between **x**_0_ and **x**_*i*_ is used:

(23) $$\begin{array}{c} d_{\text{PG}}\left(x_{0},x_{\left(i\right)}\right)=\sum_{k=0}^{i}\mu_{1}\left(x_{0},x_{\left(k\right)}\right),\;\text{for }i=\left\{0,\ldots ,n^{2}-1\right\}, \end{array}$$

where 1 ≤ *d*_PG_(**x**_0_, **x**_(*i*)_) ≤ *n*^2^, for *i*={0,…, *n*^2^ − 1}.

A fuzzy set *large*(*·*)^ℒ^ is used to represent the fuzzy variable *d*_PG_(**x**_0_, **x**_(*i*)_)*large*:

(24) $$\begin{array}{c} {\left(d_{\text{PG}}\left(x_{0},x_{\left(i\right)}\right)\right)}^{ℒ}=\mu_{2}\left(d_{\text{PG}}\left(x_{0},x_{\left(i\right)}\right)\right)\\ =-\frac{1}{{\left(n^{2}-1\right)}^{2}}\left(d_{\text{PG}}\left(x_{0},x_{\left(i\right)}\right)-1\right)\times \left(\left(d_{\text{PG}}\left(x_{0},x_{\left(i\right)}\right)-2n^{2}+1\right)\right),\;\text{for }i=\left\{0,\ldots ,n^{2}-1\right\}. \end{array}$$

In order to better distinguish between noisy and noise-free pixels, it is more appropriate in establishing peer group cardinality differences. A quadratic function is normally used as it shows sensitivity in low values of cardinality more than in the high values. In the determination of membership function, there is no need to adjust further the parameter of the membership function.

A further idea discussed in that work is to calculate the parameter *r* of the *peer group* of the filter using fuzzy logic. So, the best number of members $\tilde{r}$ corresponds to the value *r*={0,…, *n*^2^ − 1} that maximizes the certainty of the resulting expression. By using the product *T*-norm as the conjunction operator, the certainty *𝒞*_(*r*)_ of *r* that corresponds to the best number of members for *𝒫*(**x**_0_, *r*, *d*) satisfies the following fuzzy reasoning argument:

(25) $$\begin{array}{c} C_{\left(r\right)}=\mu_{1}\left\{x_{0},x_{\left(r\right)}\right\}{\left(d_{\text{PG}}\left(x_{0},x_{\left(r\right)}\right)\right)}^{ℒ}, \end{array}$$

where *𝒞*_(*r*)_ represents the certainty of “**x**_0_ is similar to **x**_(*r*)_”; *μ*_1_{**x**_0_, **x**_(*r*)_} represents the extent to which the farthest pixel in *𝒫*(**x**_0_, *r*, *d*) is similar to the center pixel **x**_0_; and (*d*_PG_(**x**_0_, **x**_(*i*)_))^ℒ^ gives the certainty of “(*d*_PG_(**x**_0_, **x**_(*r*)_)) is *large*”. The best number $\tilde{r}$ of members for *𝒫*(**x**_0_, *r*, *d*) is given by the function

(26) $$\begin{array}{c} \tilde{r}=\underset{r\in \omega }{\text{arg}\max}\text{,}\;\text{for }\omega =\left\{1,\ldots ,n^{2}-1\right\}. \end{array}$$

This reasoning is used to check for each value *r*, whether the increment from (*d*_PG_(**x**_0_, **x**_(*r* − 1)_)) to (*d*_PG_(**x**_0_, **x**_(*r*)_)) is sufficiently large to include in the fuzzy peer group. Since the proposed method allows the operator to ignore the number of clusters in the particular neighborhood, which are always the results from Fisher's linear discriminant approach, this is in its essence a statistics based algorithm for designing peer group filters.

Finally, the fuzzy peer group is formulated by a similarity fuzzy set *f𝒫*(**x**_0_, **x**_(*i*)_)=*μ*_1_({**x**_0_, **x**_(*i*)_}), with peer group members $x_{\left(0\right)},x_{\left(1\right)},\ldots ,x_{\left(\tilde{r}\right)}$.

For summarization, membership functions characterize the fuzzy sets. In a fuzzy logic system (FLS), membership functions are associated with terms that appear as the antecedents or the consequences of fuzzy rules. FLS is one of the tools used to model a multi-input, multioutput system. Type-1 membership functions have been the focus in this paper.

One important issue is the derivation of membership functions that achieve fuzzy similarity measurements of the color pixels of an image. According to [7], the rank ordering of samples approach is a good starting point. A Gaussian function may be used to describe the similarity between two color pixels; this approach is more commonly adopted mainly due to its extensive use in fuzzy ranked filters.

Another way of evaluating the similarity function is introduced by [17]. A number of *convex* membership functions for evaluating the degree of similarity have been introduced in their works. A simple linear similarity function with parameter *h* is only required to be determined, which reflects the similarity of image structure. Compared to the vector median filter (VMF) approach, the resultant filter shows enhanced performance.

Exploring color similarity measurements is discussed in [51]. It is claimed that a membership function is applied to firstly achieve color component correlation; this includes both the Euclidean distance measurements associated with each color component and the measurements of the Euclidean distance difference from different pairs of color components.

As mentioned, histogram-based approaches have been developed to also derive membership functions. One interest is to link small membership function depending on slope varieties of each selected intensity value [52]. Another approach in [26] has the following two focal points: one is to establish a membership function with adaptation to a fixed-value impulse-noise, and the other is to establish a membership function to random-value impulse-noise. In the fixed-value impulse-noise case, the extreme values are compared with mean values for noise detection. For a random-value impulse-noise, the histogram algorithm achieves parameter estimation for membership function constructions.

## 4. Fuzzy Filters' Design

If a color pixel or component is considered noisy (not noise-free), it should be filtered or smoothed proportionally. The estimated value is computed using the information of its local neighbourhood or the other color components of the filtered pixel in order to better estimate the original value while preserving edge information without introducing color artefacts.

### 4.1. Proposed L-Filter

The work carried out by [62] presents a switching rule-based filter that can be switched between the identity filter (denoted as **y**_*ξ*_) and a modified L-filter design (denoted as **y**_L_mod__). Following the detecting method, this is utilized to calculate the ideal output for the pixel's intensity and color. The suggested filter is distinguished from most L-filters because it integrates just two pixels from the vector ordered set; this significantly decreases the time required for both output calculation and coefficient training. The following is the expression for the switching scheme filter.

(27) $$\begin{array}{c} y_{i}=\left\{\begin{array}{cc} y_{\xi }, & \text{if clean,}\\ y_{{\text{L}}_{\text{mod}}}, & \text{otherwise,} \end{array}\right. \end{array}$$

where **y**_*i*_ denotes the intermediate output with index *i* in a color image, corresponding to intensity or color. The switching operation is finally carried out by a combination of the outputs between intensity |*υ*| and color *θ* with optimal magnitude and optimal direction:

(28) $$\begin{array}{c} {\tilde{y}}_{i}=\left|\upsilon_{i}\right|\theta_{i}, \end{array}$$

where

(29) $$\begin{array}{c} \left|\upsilon_{i}\right|={\left(y_{\text{R}i}^{2}+y_{\text{G}i}^{2}+y_{\text{B}i}^{2}\right)}^{1/2},\\ \theta_{i}=\cos^{-1}\left(\frac{y_{\text{R}i}\cdot y_{\text{G}i}\cdot y_{\text{B}i}}{\left|\upsilon_{i}\right|}\right), \end{array}$$

where *y*_R*i*_, *y*_R*i*_, and *y*_R*i*_ denote the red, green, and blue components of the intermediate pixel vector.

The suggested L-filter is constructed by combining two pixels from the vector median ordered set linearly.

(30) $$\begin{array}{c} y_{{\text{L}}_{\text{mod}}}=\sum_{i=1}^{2}c_{i}{\tilde{y}}_{j_{i}}. \end{array}$$

Here *c*_*i*_ corresponds to the *i* th coefficient in the vector median ordered set. The subscript *j* denotes the index of the pixel selected from the ordered set. For a *n* × *n* filter window with the center position at *C*=(*n* × *n*+1)/2, *j*_1_ will be *C* − 2 and *j*_2_ will be *C* − 1. In the calculation, the center pixel is considered to be noise from the detection result, without being included as a possible output.

The constrained least mean square (LMS) algorithm optimized the coefficients using a set of target and purposely distorted pictures supplied by the user [63]. Optimization is performed to reduce the direction and amount of the inaccuracy in the color and intensity values, respectively. For more details related to the LMS algorithm, one needs to refer to [63].

In [64], through the fuzzy model, an *l*2 − *l∞* filter has been constructed for nonuniformly sampled nonlinear systems. Compared with the classical filter (i.e., Kalman filter), the *l*2 − *l∞* filter is more applicable because the requested peak value of the estimation error for the external noise is less than a certain level that often requires to be satisfied. Hence, it shows the advantage of the fuzzy modelled filter in achieving a prescribed noise attenuation level.

While the error-diffusion dither produces a relatively high-quality image, it is computationally expensive. In [65], a new approach to error diffusion dithering through a fuzzy error diffusion algorithm is proposed. To speed up the fuzzy error diffusion process, an L-filter approach is developed by determining a fixed set of membership values. The fuzzy error diffusion algorithm is performed to achieve drastic improvements of color images quality, resulting in superior-quality dithered images and significantly lower mean squared error values (MSE).  Figure 3(c) illustrates the result of fuzzy error diffusion and compares it with the classical approaches in Figures 3(d) and 3(e) along with classical error diffusion that has been used to produce the image in Figure 3(b). The original image is given in Figure 3(a). Color impulses are observed as white dots on uniformly gray colored regions. The result of the fuzzy error diffusion algorithm is given in Figure 3(c), where fuzzy error diffusion reduces the occurrence of color impulses drastically. A significantly lower MSE value for the fuzzy error diffusion algorithm is 48.3 for Figure 3(c) versus 67.4 for Figure 3(b).

### 4.2. Fast Adaptive Similarity Filter

Considering the information associated with the central pixel, [17] proposed the design of nonlinear filters to establish similarity measures in a fast, adaptive manner on the basis of the correlation between the different image channels. The algorithm benefits from a lower computational complexity than that of the vector median filter.

Following Section 3.1.2, according to equation (9), a modified cumulative distance function *R*_*k*_ can be established:

(31) $$\begin{array}{c} R_{k}=\left\{\begin{array}{cc} -h+\sum_{j=1}^{n}\rho \left(x_{k},x_{j}\right), & \text{for }k=0,\\ \sum_{j=1}^{n}\rho \left(x_{k},x_{j}\right) & \text{for }k=1,\ldots ,n. \end{array}\right. \end{array}$$

For convenience of representation, here we relabel the center pixel as **x**_0_ in this equation. The filter construction is quite similar to the standard VMF. The major difference is the omission of the central pixel **x**_0_ when calculating **x**_*k*_, *k* > 0.

The condition for retaining the original image pixel is *R*_0_ < *R*_*k*_, *k*=1,…, *n*, which leads to the condition

(32) $$\begin{array}{c} -h+\sum_{j=1}^{n}\rho \left(x_{0},x_{j}\right)\leq \sum_{j=1}^{n}\rho \left(x_{k},x_{j}\right). \end{array}$$

That means

(33) $$\begin{array}{c} R_{0}\leq R_{k}ifh\geq \sum_{j=1}^{n}\left[\rho \left(x_{0},x_{j}\right)-\rho \left(x_{0},x_{j}\right)\right], \end{array}$$

where *k*=1,…, *n*.

This technique, which is based on the basic leave-one-out strategy, is the new algorithm's most significant feature. The central pixel is only replaced when it is really noisy; this approach aims to preserve as much as possible the original information in the images.

As is commonly known, the VMF method has the problem of replacing an excessive number of uncorrupted picture pixels. This problem is addressed in the existing filter design by specifying positive *h* values, compelling the filter to retain as many uncorrupted, original pixels as possible while still allowing for the removal of corrupted ones. Additionally, *h* may be fine-tuned further based on noise statistics and image structure.

The filtering process follows three steps. (a) The fractions of corrupted pixels are estimated. As mentioned in Section 3.1.2, it is possible to find two “close” pixels among its eight neighbors and a filtered center located pixel, according to a predefined *L*_2_ distance constant *d* and the number of pixels *m* within the distance range. Outside that distance range, the pixel is considered noisy. (b) An optimal value of *h*is found. Consequently, the constant *h* is established to the value that results in the filter changing the same proportion of pixels as the predicted noise fraction *p*.

To quickly create a filter, the well-known bisection approach may be employed [66]. This approach permits the root of an equation *g*(*x*)=0 in [a, b] to be determined, provided that *g*(*x*) is continuous and *g*(*a*)*g*(*b*) < 0. In the case considered here,

(34) $$\begin{array}{c} g\left(h\right)=\lambda \left(h\right)-p, \end{array}$$

where *λ*(*h*) is the fraction of pixels changed by the filter, depending on *h*. For the majority of standard color images, a sufficiently long interval is considered as [0, 4], where *g*(0)*g*(4) < 0. (c) Filtering of an image using the obtained optimal value of *h* is subsequently performed. The algorithm incorporates the following steps: (1) Set *r*:=*a*, *s*:=*b*. (2) Set *z* : =(*r*+*s*)/2. (3) If *g*(*z*)=0, then output $\bar{\beta }=z$ and exit. In any other case, (a) if *g*(*z*)*g*(*r*) < 0, then set *s* : =*z* and go to 2. (b) If *g*(*z*)*g*(*r*) > 0, then set *r* : =*z* and go to 2. Although the described process may be of infinite length and may not give an exact value, it provides a sufficiently good approximation of $\bar{\beta }$, after a limited number of iterations.

### 4.3. Histogram-Based Fuzzy Color Filter

Referring to histogram adaptive filtering in [54, 55], the differences between intensity values in the different components can be transformed from the unit interval into the [−(2*m*+1), +(2*m*+1)] interval for a real gray intensity distribution. We denote this as △′. The filtering procedure only processes those components that have a nonzero membership degree in the fuzzy set *noise* (i.e., for the red components *μ*_noise_(*C*_R_(*k*_1_, *k*_2_)) > 0). The filtering method distinguishes four different cases, which can be illustrated for a noisy red component pixel (*C*_R_(*k*_1_, *k*_2_)) (i.e., *μ*_noise_(*C*_R_(*k*_1_, *k*_2_))), where *y*_*R*(*k*_1_, *k*_2_)_ denotes the filtered output value.

**Case 1 .**

*μ*_noise_(*C*_G_(*k*_1_, *k*_2_)) > 0 and *μ*_noise_(*C*_B_(*k*_1_, *k*_2_) > 0 *y*_R_(*k*_1_, *k*_2_))=(∑_*k*=1_^9^(1 − *μ*_noise_(*C*_G*k*_))*C*_R*k*_/∑_*k*=1_^9^(1 − *μ*_noise_(*C*_G*k*_))).

**Case 2 .**

*μ*_noise_(*C*_G_(*k*_1_, *k*_2_))=0 and *μ*_noise_(*C*_B_(*k*_1_, *k*_2_)) > 0*y*_R_(*k*_1_, *k*_2_)=*C*_G_(*k*_1_, *k*_2_)+△_RG_′*C*(*k*_1_, *k*_2_).

**Case 3 .**

*μ*_noise_(*C*_G_(*k*_1_, *k*_2_)) > 0 and *μ*_noise_(*C*_B_(*k*_1_, *k*_2_))=0*y*_R_(*k*_1_, *k*_2_)=*C*_B_(*k*_1_, *k*_2_)+△_RB_′*C*(*k*_1_, *k*_2_).

**Case 4 .**

*μ*_noise_(*C*_G_(*k*_1_, *k*_2_))=0 and *μ*_noise_(*C*_B_(*k*_1_, *k*_2_))=0*y*_R_(*k*_1_, *k*_2_)=0.5(*C*_G_(*k*_1_, *k*_2_)+△_RG_′*C*(*k*_1_, *k*_2_))+0.5(*C*_B_(*k*_1_, *k*_2_)+△_RB_′*C*(*k*_1_, *k*_2_)).

In the first case it is possible that ∑_*k*=1_^9^(1 − *μ*_noise_(*C*_R*k*_))=0 (which is exceptional). In this situation, the output value *F*_*R*_(*k*_1_, *k*_2_) is assumed to be equal to the median of all the associated pixel intensity values.

Additionally, Fotinos et al. [67] designed a multidimensional filtering technique using fuzzy logic ideas and based on local statistics, the maximum and minimum of the histogram as parameters for signal shape description. Experimental results, conducted in true color images, show improved performance in the suppression of different types of noise and the preservation of the image details compared with other popular filtering techniques in literature, such as the arithmetic mean filter (AMF), vector median filter (VMF), the mean filter, and the fuzzy multichannel filter [68].

## 5. Fuzzy Filters in the Restoration of Medical Images and Signals

The large number of sensors and hyperspectral imaging modalities adopted in medical imaging leads to different types of noise [69, 70], which may coexist when the images are the result of data fusion procedures. Noise that is not informative may impair visual interpretation process and affect the fidelity of automated analysis source [71]. Numerous fuzzy techniques have been investigated for restoring corrupted magnetic resonance imaging (MRI) data, including those from the brain and the heart [72–77].

### 5.1. Filtering Heart MRI Data

In [72], a unique postprocessing approach is introduced via considering phase-contrast magnetic resonance imaging. Automatic vessel segmentation is accomplished using active contours [78, 79], while the segmented velocity field is filtered by applying multidimensional fuzzy adaptive vector median filtering. Accordingly, the processed MRI data is from children born with congenital single-ventricle heart abnormalities. The study demonstrates the algorithm's capability of visualizing and quantifying hemodynamics, as well as identifying patients with heart failure risks.

Random noise is introduced during segmentation as a consequence of a fuzzy vessel edge. A hybrid multichannel filter architecture is suggested to identify and replace this noise.

(35) $$\begin{array}{c} y\left(\overset{⟶}{k}\right)=\mu \left(\overset{⟶}{k}\right)x\left(\overset{⟶}{k}\right)+\left(1-\mu \left(\overset{⟶}{k}\right)\right)M\left(\overset{⟶}{k}\right), \end{array}$$

where *x* denotes the input vector, $\overset{⟶}{k}\left(k_{1},k_{2}\right)$ signifies the pixel coordinate vector, *M* is the selected filter value to replace the vector's noisy component, and *μ* denotes a continuous fuzzy membership determining the extent of *x* being a flow pixel. Vector median filtering is presented for the analysis of a segmented PC MRI dataset, a vector field having three components for each data point. Due to the physical properties of flow and noise, the parameters used to establish these rules are as follows: (i) VDH or vector direction homogeneity; (ii) DVM or the distance of the given pixel from the vector median within the interrogation window; (iii) MI or magnitude image intensity; and (iv) SD or the standard deviation of the vector field. As a result, a set of generic principles for characterizing flow and noise may be defined as follows.

- *Rule 1*. DVM is high for noise and low for flow
- *Rule 2*. VDH is low for noise and high for flow
- *Rule 3*. SD is high for noise and low for flow
- *Rule 4*. MI is low for noise and high for flow

Then, using fuzzy fusion, a membership function *μ* is assessed to estimate the chance of a pixel being noise.  Figure 5 shows an example of noise used in active contour-based segmentation. Along the vessel walls, noise vectors are readily visible inside this segmented vessel, as shown by the oval [72].

### 5.2. Filtering Brain MRI Data

Additionally, [80] included a switch mode fuzzy adaptive median filter (SMFAMF), which is used to reduce noise in MR images distorted by significant impulse (salt and pepper) noise without damaging picture edges and features. The authors next examined the same issue using a fuzzy adaptive median filter with adaptive membership parameters (FAMFAMP) [81]. It was discovered that it outperformed the SMFAMF when it came to suppressing salt-and-pepper noise and other noise of impulse type.

Bappy and Jeon [82] restored medical X-ray pictures using total variation (TV) minimisation and a hybrid median filter (HMF), with the goal of preserving edges and essential image information for accurate illness identification by doctors or radiologists. The resulting experiment demonstrates increased convergence speed and the restoration of high-quality medical X-ray pictures, with the staircase effect and spurious edges erased.

### 5.3. Filtering Multimodality Medical Images

Today there have been several medical imaging modalities, including structural modalities and functional modalities. Functional modalities include single-photon emission CT (SPECT), positron emission tomography (PET), and functional magnetic resonance imaging (fMRI) images that provide more information about functional tissues like blood flow in a vein. On the other hand, structural modalities include magnetic resonance imaging (MRI) and computed tomography (CT) that render high-resolution structural information about an organ. Each modality has its respective advantages and disadvantages.

Ullah et al. [83] coupled Sum-Modified-Laplacian (SML) algorithms and local featured fuzzy sets in the nonsubsampled Shearlet Transform (NSST) domain to develop color medical picture fusion that effectively restrains color distortion and improves visual quality. The technique involves decomposing two registered pictures of the same scene into a single Low-Frequency Subband (LFS) and numerous High-Frequency Subbands (HFS). On the LFS, the weights of each pixel are determined using Fuzzy Pixel-based fusion algorithms. To extract more meaningful information, merged HFS coefficients are chosen based on the SML coefficients of each HFS. Finally, the appropriate fused picture is obtained using inversed NSST. To evaluate performance, 256 × 256 MRI, PET, and SPECT images are picked for the fused MRI/PET and MRI/SPECT images. The obtained results demonstrate that the proposed approach is not only better in terms of contour and edge detection, visual feature recognition, and computing performance, but also in terms of quantitative parameters when compared to other state-of-the-art offered systems, such as Fuzzy Transform with uniform sinusoidal membership fusion [84], PCNN model [85, 86] for the fusion of LFS and HFS, local Laplacian filtering (LLF) [87] for image decomposition, contourlet transform (COT) [88], nonsubsampled contourlet transform (NSCT) [88], moving frame based decomposition framework (MFDF) [89], and sparse representation (SR) based approach [90].

### 5.4. Fuzzy Rule-Based Methods for Earlier Cancer Diagnosis

Currently, Fuzzy rule-based systematic approaches have been developed for early cancer diagnosis with the analysis of medical images. Mammogram images are being acquired to aid the breast cancer diagnosis of the suspected patients. Rao et al. [91] implemented fuzzy rules with minimum phases for the analysis of mammographic images that consist of 320 images coming from 160 patients with each of 1024 × 1024 resolutions. We calculate statistical metrics such as the Correct Detection Ratio (CDR), the Undersegmentation Error (USE), and the Similarity Index (SI). The suggested method gives quicker, more accurate findings that are more helpful in diagnosing and classifying aberrant tumors or masses while incurring less processing costs.

Tiwari et al. [92] defined medical entities as fuzzy sets and reasoning as rule-based systems in order to explore the likelihood of incidence of lung infection. It is regarded to be a safe and cost-effective method of treating lung disorders. Additionally, fuzzy logic implementation gives a set of approaches for obtaining dependable solutions. Kumar et al. [93] created a Combined Fuzzy-Rough-Set-Based F-Information and Water Swirl Algorithm with the goal of automating the discovery of cancer-associated genes (FRFI-WSA). There are two phases of gene selection: filtering and embedding, which are used to identify prospective genes and the most important cancer genes. The suggested technique is assessed on 9 binary and 13 multicategory cancer gene expression datasets. In the global cancer map with repeated measurements (GCM-RM) dataset, FRFI-WSA identified the 16 most significant genes linked with cancer with the fewest possible compact rules and the maximum classification accuracy of 96.45%.

For an extended application in biomedicine, Harsha and Vajpai [94] illustrate a Fuzzy Inference System that is used for the analysis and classification of electroencephalogram (EEG) signals. Statistical analysis of dynamical properties of the EEG signals is performed and the outcome of this analysis is used to create a fuzzy inference model. The final aim is to differentiate between brain states and zones they belong to, for example, healthy zone, epileptic zone, and nonepileptic zone. Encouraging results have been obtained from this pilot project. Further generalization of the rules is possible with the help of more data and inputs from neurophysiological experts.

## 6. Conclusion

This paper is focused on fuzzy filtering with type-I fuzzy reasoning, using some well-known fuzzy filter design approaches. Different fuzzy variable designs using different fuzzy rules were considered. Furthermore, different membership functions with optimized parameters were also discussed. Advances in the design of multichannel hybrid filters originally proposed in [23] have been considered, and their evolution all the way until the development of fuzzy peer group filter designs, which were introduced in 2009 [59], has been summarized. These designs have over the years been gradually simplified and evolved to variants requiring less computational complexity. What must be stressed out, however, is that these ideas form an important intellectual scaffolding for further developments in this field. Finally, within the context of biomedical imaging applications, what is particularly attractive is that these filters can be adapted to provide resilient energy-to-peak filter designs for each pixel or voxel, when nonlinearities in the image need to be preserved after assuming a Takagi–Sugeno fuzzy model where the designed filter is assumed to have additive gain variations [95]. Furthermore, these designs complement well existing wavelet parametrizations with adaptive filtering [96, 97], so it is thus envisaged that the fuzzy filtering techniques may also be soon applied to wavelet parametrizations (at different decomposition levels) so as to significantly improve filtering and signal reconstruction. Fuzzy filters are especially promising in MRI image denoising and have applications to hyperspectral imaging, and in cases when combining terahertz (THz) imaging with images from different parts of the electromagnetic spectrum (e.g., near infrared, visible, or ultraviolet parts of the spectrum). In addition, they have applications in magnetic resonance imaging (MRI) [73, 75, 97–103], retinal fundus photography [104, 105], face recognition [106], and video analysis [107].

Furthermore, they have important applications in optical coherence tomography and fundus imaging [108], in electroencephalogram (EEG) analysis [109, 110], and in other tomographic applications (e.g., in 3-dimensional reconstruction of brain images [111] or X-ray computed axial tomography [112] or ultrasound [113, 114]). The collective discussion of the various fuzzy filtering approaches in this article should lead to a better understanding of what has been achieved so far by the fuzzy filtering community and provides some further directions for research. From an applications perspective, an adaptation and evaluation of these algorithms for the different biomedical imaging modalities mentioned is urgently needed.

## Figures and Tables

**Figure 1:** (a) Illustration of the neighborhood of a central pixel (**k**) within a 3 × 3 window demonstrated by a thick solid black line. (b) Illustration of centers for the calculation of the basic and related gradient values in the NW-direction and an example of an edge related to the local area inside the window. The latter is represented by a thick dash line.

**Figure 2:** Illustration of the membership function *large*.

**Figure 3:** (a) Original image, (b) classical error diffusion (MSE = 67.4), (c) fuzzy error diffusion (MSE = 48.3), (d) L-filter with common memberships (MSE = 50.5), (e) L-filter with four fixed membership values (0.82, 0.14, 0.03, and 0.01) (MSE = 49.8), and (f) L-filter with two fixed membership values (0.85 and 0.15) (MSE = 51.8) [65].

**Figure 4:** From top left to bottom right, (a) a part of the original colored Lena image and (b) the part corrupted with 20% salt-and-pepper noise (PSNR: 12.29). (c) After the proposed HFC (PSNR: 46.84). (d) After the FIDRM (PSNR: 34.97). (e) After the AWFM (PSNR: 30.58). (f) After the HAF (PSNR: 29.19). (g) After the DSFIRE (PSNR: 30.75). (h) After the TSM (PSNR: 28.05). (i) After the VMF (PSNR: 29.12) [26].

**Figure 5:** An example of noise being embedded into active contour-based segmentation [72].
